# Measures of Adiposity and Risk of Testing Positive for SARS-CoV-2 in the UK Biobank Study

**DOI:** 10.1155/2021/8837319

**Published:** 2021-01-22

**Authors:** Rebecca A. G. Christensen, Shelby L. Sturrock, Jasleen Arneja, Jennifer D. Brooks

**Affiliations:** Dalla Lana School of Public Health, University of Toronto, Toronto, ON, Canada

## Abstract

**Objective:**

To assess if body mass index (BMI) and high waist circumference (HWC) are associated with testing positive for the severe acute respiratory syndrome coronavirus 2 (SARS-CoV-2).

**Methods:**

9,386 UK Biobank study participants tested for SARS-CoV-2 from March 16^th^ 2020 to June 29^th^ 2020 were analyzed. A forward model building approach was used to estimate adjusted risk ratios (RR) and 95% confidence intervals (95% CI). Analyses were stratified by age due to a significant first-order interaction between age and HWC.

**Results:**

Approximately 17% (*n* = 1,577) of participants tested positive for SARS-CoV-2. BMI category had a linear association with testing positive for SARS-CoV-2 among participants <65 years (*RR* = 1.09, 95% CI 1.02–1.17). For participants ≥65 years, only obesity class II (*RR* = 1.38, 95% CI 1.10–1.74) had a significantly greater risk of testing positive for SARS-CoV-2 than those who were underweight/normal weight. While HWC was not associated with testing positive for SARS-CoV-2 in those <65 years, having an HWC was associated with an increased risk of testing positive for SARS-CoV-2 in participants ≥65 years (*RR* = 1.12, 95% CI 1.00–1.27).

**Conclusion:**

The associations of BMI and HWC with testing positive for SARS-CoV-2 differed by age. Notably, HWC was associated with testing positive in those ≥65 years, but not those who were younger, independent of BMI. This suggests that measures of adiposity in addition to BMI may be used to identify older individuals at greater risk of testing positive for SARS-CoV-2.

## 1. Introduction

Increased adiposity, as assessed by body mass index (BMI) [1, 2] and waist circumference [1, 2], is a well-established risk factor for several chronic conditions, including those associated with increased severe acute respiratory syndrome coronavirus 2 (SARS-CoV-2) severity, such as diabetes [3], hypertension [3], chronic lung disease [3], and cancer [4]. Furthermore, excess weight has been shown to be a risk factor for SARS-CoV-2-related morbidity and mortality [5–7]. Emerging evidence suggests excess weight (i.e., BMI [8–11], waist circumference [9], waist-to-hip ratio [11], and visceral adiposity [12]) may also be associated with an increased risk of testing positive for SARS-CoV-2. Here, we examine if measures of adiposity, BMI, and high waist circumference (HWC) are associated with testing positive for SARS-CoV-2 among participants in the UK Biobank (UKB) study.

## 2. Methods

This research has been conducted using the UK Biobank (UKB) Resource [13]. The UKB is a convenience-based sample of approximately 500,000 adults aged 40–69 years [13]. Participants were recruited from 2006 to 2010 and have been followed prospectively through linkage to administrative health databases. Recruitment and data collection procedures are described elsewhere [13].

Between March 16 and June 29, 2020, a total of 14,439 SARS-CoV-2 tests were performed on 9,494 UKB participants [14]. Participants included in this study were tested in both community and in-patient settings. The majority of tests were nasal or throat swabs, and all underwent PCR testing [14]. Individuals with at least one positive test were classified as positive for SARS-CoV-2 (yes/no). Participants were excluded if they were missing data on BMI (*n* = 103) or waist circumference (*n* = 5), leaving 9,386 for the current analysis.

BMI and waist circumference were measured at baseline by trained technicians. BMI was categorized as underweight/normal weight (<25 kg/m^2^), overweight (25 to <30 kg/m^2^), obesity class I (30 to <35 kg/m^2^), obesity class II (35 to <40 kg/m^2^), and obesity class III (≥40 kg/m^2^) [15]. HWC (yes/no) was categorized using sex- and BMI-specific thresholds [16] (Table 1). Current age was derived using month and year of birth and month of testing.

Sociodemographic characteristics (e.g., ethnicity and education), lifestyle risk factors (e.g., smoking and alcohol use frequency), and medical history (e.g., cancer and respiratory disorders) were self-reported at baseline. Medical conditions developed over the course of follow-up were accounted for using ICD-10 codes from linked administrative data (in-patient hospital records and cancer registry data) (Table 2). The following variables were evaluated as confounders: age at SARS-CoV-2 testing, sex (male/female), education (secondary/postsecondary/missing), and alcohol use frequency (never/special occasions only/one to three times a month/once to twice a week/three or four times a week/missing) at baseline, as well as chronic conditions (ascertained at baseline and prospectively through administrative databases).

### 2.1. Statistical Analysis

Standardized differences (SD) were used to detect clinically relevant (i.e., ≥10% [17]) differences between the general UKB population and the subsample tested for SARS-CoV-2.

Multivariable Poisson regression models with robust variance estimators were used to estimate unadjusted and adjusted risk ratios (RR) and 95% confidence intervals (CI) for the association of BMI category (as a nominal or ordinal variable) and HWC (yes/no) and risk of testing positive for SARS-CoV-2 [18]. A forward model building approach [19] was used to identify important confounders.

Effect measure modification was assessed by including the first-order interaction between each risk factor retained in the model and the measures of adiposity and stratified estimates produced where indicated. All analyses were conducted using SAS version 9.4; results were considered statistically significant at an alpha of 0.05.

## 3. Results

Among UKB participants tested for SARS-CoV-2, the median age was 69 years (interquartile range: 61–75). Almost half of the sample was male (*n* = 4,564, 48.6%), the average BMI was 28.3 ± 5.3 kg/m^2^, and 30.6% (*n* = 2,868) of participants had a HWC (Table 2). There were some clinically meaningful differences in participants tested for SARS-CoV-2 and the general UKB sample. Specifically, participants tested for SARS-CoV-2 had a higher BMI (28.3 ± 5.3 versus 27.4 ± 4.8 kg/m^2^, SD: 17.4%) and a larger waist circumference (93.3 ± 14.3 versus 90.3 ± 13.5 cm, SD: 21.2%) than the full UKB cohort. In addition, participants tested for SARS-CoV-2 reported a significantly higher burden of chronic conditions (SD: 22.1%), with more than 87% (*n* = 8,198) reporting at least one chronic condition other than obesity, compared to 79% (*n* = 397,705) in the overall UKB sample. Of the 9,386 adults tested for SARS-CoV-2, 1,577 (16.8%) tested positive.

Demographic variables retained within the model include age, sex, race, and education. Lifestyle factors (i.e., smoking and alcohol use) and three chronic conditions (i.e., whole organ transplant, inflammatory disease of the central nervous system, and liver disease) were also included in the final multivariable model in addition to BMI category and HWC. Effect measure modification was demonstrated by a significant first-order interaction between age and HWC (*P*=0.0199). Therefore, all models were stratified by age.

BMI was positively associated with testing positive in participants <65 years of age (*RR* = 1.09, 95% CI 1.02 to 1.17 per category increase in BMI). In participants ≥65 years of age, there was no evidence of a linear trend (*RR* = 1.05, 95% CI 0.99 to 1.11 per category increase in BMI). Instead, only participants with obesity class II compared to individuals with underweight or normal weight were at a significantly increased risk for testing positive for SARS-CoV-2 in this group (*RR* = 1.38, 95% CI 1.10 to 1.74). Participants with obesity class III did not exhibit any increased risk (*RR* = 0.99, 95% CI 0.70 to 1.40). In individuals <65 years of age, HWC was not significantly associated with testing positive for SARS-CoV-2 (RR = 0.93, 95% CI 0.77 to 1.12) (Table 3). Conversely, in those ≥65 years of age, having HWC was associated with 1.12 (95% CI 1.00 to 1.27) times the risk of testing positive for SARS-CoV-2.

## 4. Discussion

This is the first study to show that the association between adiposity and testing positive for SARS-CoV-2 varies by age. Specifically, while the risk of testing positive for SARS-CoV-2 increased with increasing BMI category among participants <65 years of age; only obesity class II was statistically significantly associated with increased risk among participants ≥65. This is consistent with research outside the SARS-CoV-2 setting, suggesting that the association between weight and health outcomes differs by age. For example, having a moderately higher weight is associated with positive health outcomes (e.g., decreased premature mortality) in older populations [20].

It is unclear why obesity class III was not significantly associated with testing positive for SARS-CoV-2 in older adults in our study. Two studies [10, 11], which also used the UKB study, observed a linear association between BMI and testing positive for SARS-CoV-2, and one study reported there was no effect of older age [10]. However, both studies [10, 11] examined severe SARS-CoV-2 infection (i.e., patients tested in-hospital), while we included participants tested both in the community and in-patient settings. Thus, these differences could be due to the fact we included all individuals who tested positive for SARS-CoV-2 and thereby including individuals with both mild and severe diseases. While lack of association for individuals with an obesity class III could be attributed, in part, to survivorship bias, it could also be related to having fewer opportunities for exposure to/contact with individuals infected with SARS-CoV-2 due to poorer health or because they were following the government recommendations for clinically vulnerable populations to remain home (a.k.a., shielding) [21]. Specifically, participants with obesity class III had a median of ten chronic conditions (median (IQR): 10.0 (7.0 to 13.0) chronic conditions), and 98.2% of these participants had at least one chronic condition other than obesity.

Previous research has identified that waist-to-hip ratio (a measure of central adiposity) [11] and visceral adiposity [12] increase the risk of severe SARS-CoV-2 infections, defined as hospitalization, intensive care admissions, and mechanical ventilation. A positive association between waist circumference (continuous) and testing positive for [9] and dying from [22] SARS-CoV-2 has also been shown; however, these analyses did not adjust for BMI [9, 22]. These two measures of adiposity are highly correlated because waist circumference increases with BMI. Thus, assessing waist circumference without simultaneously accounting for BMI could be considered equivalent to simply assessing BMI. Ours is the first study to examine waist circumference independent of BMI. Specifically, we used BMI-specific HWC thresholds and observed that HWC was an independent risk factor for SARS-CoV-2 in individuals ≥65 years of age, but not for those younger. Findings from the current study build on this existing literature and suggest that measures of central adiposity, such as HWC, are associated with a greater risk of testing positive for SARS-CoV-2 for a given BMI in older individuals.

A main strength of this study is that our main exposures are validated measures assessed by trained technicians. SARS-CoV-2 testing took place in community and in-patient settings, capturing mild and severe disease. Another strength is the consistency of some of our findings regarding established SARS-CoV-2 risk factors. Several authors have identified being a visible minority [8, 23–26] to be risk factors for SARS-CoV-2 incidence or severity. Consistent with these findings, individuals who identified as Black or Asian were at a significantly greater risk of testing positive for SARS-CoV-2 than white participants.

One limitation is the long duration (i.e., 10–14 years) between baseline assessment and SARS-CoV-2 testing. Other papers using the same dataset have reported a high correlation between available repeat measurements of BMI (Pearson's *r* = 0.9) [11, 22]. Nonetheless, to address the potential misclassification bias time between measurements that may have introduced, we categorized our main exposure (BMI). Due to lack of out-patient clinic data, we also likely underestimated the burden of comorbidities. Another potential limitation is that excess weight increases the risk of a broad range of respiratory infections and symptoms of other endemic diseases (e.g., the flu) [27]. As testing was initially primarily restricted to those with nonspecific symptoms of respiratory infection, conditions that increase susceptibility to other viruses are overrepresented in the tested population. While 63% of adults in England have overweight or obesity [28], over 72% of UKB participants tested for SARS-CoV-2 had excess weight; thus, the reported effect size could be underestimated. Further differences between those tested for SARS-CoV-2 and the general UK populations are likely due to testing guidelines (that allocate resources to high-risk groups). Although our findings may not be generalizable to the general public, they should be generalizable to those who are prioritized for SARS-CoV-2 testing. Finally, race-specific BMI thresholds have been proposed [29] and, while not currently endorsed by the World Health Organization [29], have been used in other SARS-CoV-2 studies [7]. We were unable to use race-specific BMI thresholds in this current study as we were interested in examining the effects of severe obesity (i.e., obesity classes II and III), and to our knowledge, no race-specific thresholds or any BMI-specific waist circumference thresholds exist for severe obesity.

In summary, we observed age-specific associations between measures of adiposity and testing positive for SARS-CoV-2. There was a greater burden of morbidity in our population than would be expected in the general population which may limit the generalizability. Nonetheless, findings suggest that other measures of adiposity (i.e., HWC) may be used in addition to BMI to identify older individuals at increased risk of testing positive for SARS-CoV-2.

## Figures and Tables

**Table 1:** Sex- and BMI-specific thresholds for HWC.

	Men	Women
Underweight or normal weight	≥90 cm	≥80 cm
Overweight	≥100 cm	≥90 cm
Obesity class I	≥110 cm	≥105 cm
Obesity classes II and III	≥125 cm	≥115 cm

**Table 2:** Characteristics of the individuals tested for SARS-CoV-2 compared to the full UKB population.

Variable	Whole UKB population	Tested for SARS-CoV-2	Standardized differences
Total number tested for SARS-CoV-2	502,505	9,386	—
Demographics			
Age, median (IQR)	69 (61 to 75)	71 (62 to 77)	**17.7**
Weight in kg (mean ± std)	78.1 ± 15.9	80.6 ± 17.1	**15.2**
Male, *n* (%)	229,122 (45.6)	4,564 (48.6)	6.1

Race, *n* (%)			
White	473,594 (94.3)	8,634 (92.0)	−8.6
Asian^a^	11,456 (2.3)	255 (2.7)	2.8
Black	8,061 (1.6)	263 (2.8)	8.2
Mixed	2,958 (0.6)	69 (0.7)	1.7
Missing	6,436 (1.3)	165 (1.8)	3.9

Education, *n* (%)			
Less than postsecondary^b^	108,937 (21.7)	1,866 (19.9)	−3.3
Postsecondary^c^ (*n* (%))	300,005 (59.7)	5,218 (55.6)	−8.3
Missing^d^ (*n* (%))	93,563 (18.6)	2,302 (24.5)	14.4

Anthropometric measures			
Body mass index in kg/m^2^, mean ± std	27.4 ± 4.8	28.3 ± 5.3	17.4
Body mass index category, *n* (%)			
Underweight/normal weight	165,072 (33.1)	2,590 (27.6)	−**11.5**
Overweight	212,155 (42.5)	3,888 (41.4)	−1.6
Obesity class I	87,574 (17.5)	1,930 (20.6)	8.0
Obesity class II	24,998 (5.0)	659 (7.0)	8.6
Obesity class III	9,705 (1.9)	319 (3.4)	9.1
Waist circumference in cm, mean ± std	90.3 ± 13.5	93.3 ± 14.3	**21.2**
HWC (yes)	127,112 (25.4)	2,868 (30.6)	**11.5**

Lifestyle risk factors			
Smoke status, *n* (%)			
Never	201,734 (40.2)	3,404 (36.3)	7.2
Current	52,978 (10.5)	1,207 (12.9)	2.9
Previous	245,688 (48.9)	4,726 (50.4)	−8.0
Missing	2,105 (0.4)	49 (0.5)	1.5

Alcohol use frequency, *n* (%)			
Daily	101,769 (20.3)	1,848 (19.7)	−1.4
Three or four times a week	115,438 (23.0)	1,889 (20.1)	−6.9
Once or twice a week	129,292 (25.7)	2,276 (24.3)	−3.4
One to three times a month	55,855 (11.1)	1,065 (11.4)	0.7
Special occasions only	58,008 (11.5)	1,268 (13.5)	5.9
Never	40,641 (8.1)	1,006 (10.7)	9.0
Missing	1,502 (0.3)	34 (0.4)	1.1

Chronic conditions			
Immune system disorders, *n* (%)			
Whole organ transplant^e^	22,665 (4.5)	567 (6.0)	6.9
HIV/AIDS	23,950 (4.8)	813 (8.7)	**15.6**
Inflammatory disease of the CNS	3,232 (0.6)	91 (1.0)	3.6
Other immune system disorders^f^	101,217 (20.1)	2,556 (27.2)	**16.7**

Cardiovascular disease, *n* (%)			
Hypertension	177,751 (35.4)	4,484 (47.8)	**25.4**
Cholesterol disease	145,800 (29.0)	3,984 (42.5)	**28.3**
Ischaemic heart disease	137,546 (27.4)	3,995 (42.6)	**32.3**
Pulmonary heart disease	173,408 (34.5)	4,667 (49.7)	**31.2**
Other forms of heart disease	148,611 (29.6)	4,321 (45.1)	**32.5**
Cerebrovascular disease	150,057 (29.9)	4,278 (45.6)	**32.9**

Respiratory disorders, *n* (%)			
Bronchitis/emphysema	92,861 (18.5)	2,682 (28.6)	**24.0**
COPD	87,445 (17.4)	2,590 (27.6)	**24.6**
Asthma	114,266 (22.7)	2,983 (31.8)	**20.4**
Other respiratory disorders^g^	99,710 (19.8)	2,807 (29.9)	**23.5**
Liver disease^h^, *n*(%)	206,824 (41.2)	5,022 (53.5)	**24.9**
Kidney failure, *n*(%)	82,388 (16.4)	2,065 (22.0)	**14.3**
Diabetes, *n*(%)	60,106 (12.0)	1,866 (19.9)	**21.8**
Cancer, *n*(%)	81,944 (16.3)	1,857 (19.8)	9.1
Has ≥ 1 chronic disease, *n*(%)	397,705 (79.1)	8,198 (87.3)	**22.1**
Number of chronic diseases, median (IQR)	2 (1 to 6)	5 (1 to 9)	**41.1**

IQR: interquartile range; std: standard deviation; %, percent; HWC: high waist circumference; CNS: central nervous system; COPD: chronic obstructive pulmonary disorder. Continuous variables are present as mean ± standard deviation or median (interquartile range), and categorical variables are present as frequency (prevalence). ^a^Indian, Pakistani, Bangladeshi, Chinese, other Asians, mixed, others, and missing. ^b^CSEs or equivalent, O levels/GCSEs or equivalent, and A levels/AS levels or equivalent. ^c^Vocational school, college or university degree, and other professional qualifications. ^d^None of the above and missing. ^e^Includes the lung, kidney, liver, and pancreas. ^f^Includes lupus and certain disorders involving immune mechanisms. ^g^Includes other diseases of the upper respiratory tract, lung disease due to external agents, other respiratory diseases affecting the interstitium, other diseases of the pleura, and other diseases of the respiratory system. ^h^Includes alcoholic liver disease, hepatic failure, chronic hepatitis, fibrosis and cirrhosis of the liver, other inflammatory liver diseases, and other diseases of the liver. Standardized differences in bold represent clinically meaningful differences between groups.

**Table 3:** Association between measures of adiposity and testing positive for SARS-CoV-2 overall and stratified by older age.

Variable	Full population^†^	Under 65 years^†‡^ (range 50–64)	65 years of age or older^†^ (range 65–84)
Total number tested for SARS-CoV-2, *n* (%)	9,386	2,872 (30.6)	6,514 (69.4)
Tested positive for SARS-CoV-2, *n* (%)	1,577 (16.8)	598 (20.8)	979 (15.0)

Demographics			
Male	1.23 (1.12 to 1.34) ^*∗*^	1.14 (0.98 to 1.32)	1.29 (1.14 to 1.46) ^*∗*^
Race			
White	Ref	Ref	Ref
Asian	1.60 (1.30 to 1.97) ^*∗*^	1.79 (1.35 to 2.36) ^*∗*^	1.56 (1.13 to 2.15) ^*∗*^
Black	1.74 (1.44 to 2.10) ^*∗*^	1.64 (1.28 to 2.10) ^*∗*^	1.89 (1.43 to 2.51) ^*∗*^
Mixed	1.01 (0.60 to 1.70)	0.63 (0.28 to 1.40)	1.82 (0.96 to 3.44)
Missing	1.25 (0.93 to 1.67)	1.34 (0.92 to 1.96)	1.30 (0.82 to 2.06)

Anthropometric measures			
Body mass index categories (continuous)	1.06 (1.02 to 1.11) ^*∗*^	1.09 (1.02 to 1.17) ^*∗*^	1.05 (0.99 to 1.11)
Body mass index categories			
Underweight/normal weight	Ref	Ref	Ref
Overweight	1.14 (1.01 to 1.28) ^*∗*^	1.17 (0.98 to 1.39)	1.12 (0.96 to 1.31)
Obesity class I	1.12 (0.98 to 1.28)	1.10 (0.88 to 1.36)	1.13 (0.95 to 1.35)
Obesity class II	1.35 (1.13 to 1.61) ^*∗*^	1.35 (1.03 to 1.78) ^*∗*^	1.38 (1.10 to 1.74) ^*∗*^
Obesity class III	1.15 (0.89 to 1.48)	1.61 (1.12 to 2.32) ^*∗*^	0.99 (0.70 to 1.40)
HWC	1.06 (0.96 to 1.17)	0.93 (0.77 to 1.12)	1.12 (1.00 to 1.27) ^*∗*^

^*∗*^Statistically significant (*P* < 0.05). ^†^Estimates are adjusted for age at testing, race, education, body mass index categories, HWC, smoking status, alcohol use, whole organ transplant, inflammatory disease of the central nervous system, and liver disease. ^‡^9 excluded for missing alcohol information preventing convergence.

## Data Availability

Data are owned by the UK Biobank. Researchers may contact the UK Biobank directly in order to access the data.
